The article "Identification of Candidate Therapeutic Target Genes and Profiling of Tumor-Infiltrating Immune Cells in Pancreatic Cancer via Integrated Transcriptomic Analysis" was retracted in 2023. Reasons: suspected computer-generated content; unreliable results or conclusions; concerns about the data; concerns about the results or conclusions.

# Identification of Candidate Therapeutic Target Genes and Profiling of Tumor-Infiltrating Immune Cells in Pancreatic Cancer via Integrated Transcriptomic Analysis

**DOI:** 10.1155/2022/3839480

**Published:** 2022-08-23

**Authors:** Wei Ding, Yuxu Wang, Yongbiao Ma, Li Lin, Manjiang Li

**Affiliations:** Department of Hepatobiliary & Pancreatic Surgery, Weifang People's Hospital, No. 151 of Guangwen Street, Weifang, 261041 Shandong Province, China

## Abstract

Pancreatic cancer (PC) has a dismal prognosis despite advancing scientific and technological knowledge. The exploration of novel genes is critical to improving current therapeutic measures. This research is aimed at selecting hub genes that can act as candidate therapeutic target genes and as prognostic biomarkers in PC. Gene expression profiles of datasets GSE101448, GSE15471, and GSE62452 were extracted from the GEO database. The “limma” package was performed to select differentially expressed genes (DEGs) between PC and normal tissue samples in each dataset. Robust rank aggregation (RRA) algorithm was conducted to integrate multiple expression profiles and identify robust DEGs. GO analysis and KEGG analysis were conducted to identify the functional correlation of the DEGs. The CIBERSORT algorithm was conducted to estimate the immune cell composition of each tissue sample. STRING and Cytoscape were used to establish the protein-protein interaction (PPI) network. The cytoHubba plugin in Cytoscape was performed to identify hub genes. Survival analysis based on hub gene expression was performed with clinical information from TCGA database. 566 robust DEGs (338 upregulated genes and 226 downregulated genes) were identified. Tumor tissue had a higher infiltration of resting dendritic cells and tumor-associated macrophages (TAM), including M0, M1, and M2 macrophages, while infiltration levels of B memory cells, plasma cells, T cells CD8, T follicular helper cells, and NK cells in normal tissue were relatively higher. GO terms and KEGG pathway analysis results revealed enrichment in tumor-associated pathways, including the extracellular matrix organization, cell−substrate adhesion cytokine−cytokine receptor interaction, calcium signaling pathway, and glycine, serine, and threonine metabolism, to name a few. Finally, FN1, MSLN, PLAU, and VCAN were selected as hub genes. High expression of FN1, MSLN, PLAU, and VCAN in PC significantly correlated with poor prognosis. Integrated transcriptomic analysis was used to provide new insights into PC pathogenesis. FN1, MSLN, PLAU, and VCAN may be considered as novel biomarkers of PC.

## 1. Introduction

PC is one of the deadliest malignant tumors. The global incidence of PC in 2020 was 495,773, with 466,003 reported deaths [1]. Current treatment methods for PC mainly emphasize surgery, chemotherapy [2], radiotherapy, and immunotherapy. Although surgical resection is considered potentially curative, most pancreatic cancers are difficult to diagnose in the early stages. Reports suggest that only 15% to 20% of PC patients are suitable for surgical resection, and most patients relapse within one year after surgery [3]. Notwithstanding that advancements in medical technologies have improved the ability of clinicians to detect, diagnose, and treat, a 5-year survival rate of 8% [4] has been reported, emphasizing the need to improve patient prognosis. Therefore, to improve the current management of PC, it is paramount to find new therapeutic targets and new prognostic biomarkers.

The article "Identification of Candidate Therapeutic Target Genes and Profiling of Tumor-Infiltrating Immune Cells in Pancreatic Cancer via Integrated Transcriptomic Analysis" was retracted in 2023. Reasons: suspected computer-generated content; unreliable results or conclusions; concerns about the data; concerns about the results or conclusions.

With extensive developments made in computer science and bioinformatics analysis, public databases including GEO and TCGA database have been increasingly used for enrichment analysis and identification of DEGs between tumor and normal tissue. A study by Deng et al. found 12 genes (GPR84, IL11, PTGIS, MMP7, and MMP12, to name a few) related to survival in hepatocellular carcinoma [5]. Potential prognostic markers related to breast cancer have been reported by Wang et al. [6]. Major shortcomings of these studies include the small sample size, single dataset analysis, and heterogeneity in experimental conditions, leading to biased results. In this study, RRA algorithm was used to obtain significant DEGs. This method minimizes bias, errors, and inconsistencies between datasets and is a powerful means of screening novel prognostic genes.

Several studies have suggested that tumor microenvironment is related to tumor progression and patient survival outcomes in recent years [7]. More and more evidences show that tumor microenvironment has clinic pathological significance in predicting the effect of treatment [8, 9]. Therefore, it is possible to speculate that the changes in the tumor microenvironment, especially the different infiltration of tumor immune cells in normal tissue and tumor tissue, are one of the causes of pancreatic cancer. In the current study, we downloaded 3 datasets (GSE101448, GSE15471, and GSE62452) from the GEO database. We used the “limma software” package of R to determine the DEGs of each database. Merging of DEGs from 3 datasets was conducted using the RRA method. The functional role of robust DEGs was analyzed using enrichment analyses. Immune cell infiltration was estimated using CIBERSORT software. The PPI network was then created via a string database. The cytoHubba plugin was performed to screen hub genes via the PPI network. Survival analysis based on hub gene expression was performed with clinical information from TCGA database.

The article "Identification of Candidate Therapeutic Target Genes and Profiling of Tumor-Infiltrating Immune Cells in Pancreatic Cancer via Integrated Transcriptomic Analysis" was retracted in 2023. Reasons: suspected computer-generated content; unreliable results or conclusions; concerns about the data; concerns about the results or conclusions.

## 2. Methods

### 2.1. Data Collection and Data Processing

Three RNA-sequence files of PC were extracted from the GEO database (https://www.ncbi.nlm.nih.gov/geo/), including GSE101448 (18 tumor and 13 nontumor tissue samples), GSE15471 (36 tumor and 36 nontumor tissue samples), and GSE62452 (69 tumor and 61 nontumor tissue samples) based on the following criteria: (1) entry type, (2) gene array expression profiling based on study type, (3) Homo sapiens, (4) sample size more than 30, and (5) tumor tissue and adjacent normal tissue. We downloaded the expression matrix files and corresponding platform annotation files of the three datasets. Perl language was used to map the microarray probe data to gene symbols. “limma” software package of R was performed to select DEGs between PC and normal tissue samples in each gene expression dataset. Genes with |log_2_ fold change (FC)| > 1 and adjusted *p* < 0.05 were considered as significant DEGs.

### 2.2. Identification of Robust DEGs

Before RRA analysis, each dataset's upregulated and downregulated genes were ranked according to the logFC value. The “robust rank aggregation” R package merged DEGs from three datasets to obtain robust DEGs. Genes with |log_2_ fold change (FC)| > 1 and *p* value < 0.05 were considered as significant. A higher-ranked gene was associated with a smaller *p* value.

### 2.3. Functional Enrichment Analysis

To identify the functional roles of the robust DEGs indicated above, GO enrichment results of BP, CC, and MF were obtained using the R package “clusterProfiler.” The KEGG pathway analysis of robust DEGs was also conducted using the R package. *p* < 0.05 was considered to be statistically significant.

### 2.4. Immune Cell Infiltration

We used the *CIBERSORT algorithm* to calculate the immune composition of each tissue sample [10], with the cutoff criteria of *p* < 0.05.

### 2.5. Creation of PPI Network and Module Analysis

The PPI network of robust DEGs was created with the following method. First, the robust DEGs were uploaded to STRING [11]. Then, protein interactions with a confidence score > 0.7 were extracted from STRING and disconnected nodes were hidden from the network. The visualization of the PPI network was conducted by Cytoscape software [12]. The Cytoscape plugin MCODE was performed to select the meaningful modules from the PPI network.

### 2.6. Hub Gene Identification

To explore and screen hub genes from the PPI network, we used Cytoscape. The Cytoscape plugin cytoHubba can perform operations on several topological analysis algorithms. Hub genes were identified from these algorithms [13].

The article "Identification of Candidate Therapeutic Target Genes and Profiling of Tumor-Infiltrating Immune Cells in Pancreatic Cancer via Integrated Transcriptomic Analysis" was retracted in 2023. Reasons: suspected computer-generated content; unreliable results or conclusions; concerns about the data; concerns about the results or conclusions.

### 2.7. The Relationship between Hub Genes and Prognosis

The RNA sequence and clinical data of 178 PC samples and 4 healthy samples were extracted from TCGA database (https://portal.gdc.cancer.gov/). “Survival” and “survminer” packages were performed to explore prognosis of PC patients. The visualization of K-M plot was performed via the K-M method.

## 3. Results

### 3.1. DEG Screening

Figure 1 displays the study workflow. We used the “limma” software package of R to select for DEGs in each dataset. The selection criterion was set as |log_2_ fold change (FC)| > 1 and adjusted *p* < 0.05. In dataset GSE101448, a total of 1700 genes were significantly expressed, including 903 upregulated and 797 downregulated genes. In dataset GSE15471, a total of 919 genes were significant, including 709 upregulated and 210 downregulated genes. Finally, in dataset GSE62452, a total of 285 genes were significantly expressed, including 174 upregulated and 111 downregulated genes. Next, we used the RRA method to merge DEGs from 3 datasets. Finally, robust DEGs consisting of 338 upregulated and 226 downregulated genes were identified (Supplementary Table S1). Heat maps were generated to visualize the distribution of different genes in each dataset, and a heat map was generated to visualize the top 20 upregulated and downregulated robust DEGs (Figures 2(a)–2(d)).

### 3.2. GO and KEGG Analysis

GO enrichment analysis is used to annotate the degree of gene function terms in DEGs, which include BP, CC, and MF. The top 10 GO terms are displayed in Figures 3(a)–3(d).

GO annotation for BP included the extracellular structure and matrix organization, cell−substrate adhesion, and negative regulation of endopeptidase and peptidase activity; the CC consisted of collagen-containing extracellular matrix, endoplasmic reticulum lumen, apical part of cell, apical plasma membrane, and extracellular matrix component, while the MF involved the extracellular matrix structural constituent, glycosaminoglycan binding, serine-type peptidase activity, serine hydrolase activity, and endopeptidase regulator activity (Supplementary Table S2). GO enrichment analysis thus revealed that the robust genes were mainly related to the extracellular matrix (ECM) and could play a vital function in tumorigenesis.

KEGG pathway analysis (Supplementary Table S3) showed significant enrichment in the following pathways: cytokine−cytokine receptor interaction, calcium signaling pathway, glycine, serine, and threonine metabolism, cysteine and methionine metabolism, HIF-1 signaling pathway, PPAR signaling pathway, and metabolism of xenobiotics by cytochrome P450 (Figures 3(e)–3(h)). The enrichment analysis revealed that the robust genes were mainly related to the extracellular matrix (ECM) and change of metabolic-related pathway, which could play a vital function in tumorigenesis.

The article "Identification of Candidate Therapeutic Target Genes and Profiling of Tumor-Infiltrating Immune Cells in Pancreatic Cancer via Integrated Transcriptomic Analysis" was retracted in 2023. Reasons: suspected computer-generated content; unreliable results or conclusions; concerns about the data; concerns about the results or conclusions.

### 3.3. Immune Cell Infiltration

We use the CIBERSORT method to predict the infiltration of immune cells, as shown in Figure 4(a). As seen from the visualized heat map, compared with normal tissues, tumor tissue had a higher infiltration of resting dendritic cells and TAM (including M0, M1, and M2 macrophages). Interestingly, in normal tissue samples, B memory cells, plasma cells, CD8 T cells, T follicular helper cells, and NK cells were relatively high (Figures 4(b) and 4(c)).

### 3.4. PPI Network Creation and Module Analysis

We made the PPI network of a total of 345 nodes, and 1082 protein pairs were obtained with a combined score > 0.7 (Figure 5(a)). In total, one module with score > 15 was selected by MCODE, of which the largest connected master network contains 30 nodes and 224 edges including 28 upregulated and 2 downregulated genes (Figure 5(b)).

### 3.5. Core Gene Selection

cytoHubba, a plugin of Cytoscape, exerts different topological methods, such as maximum neighborhood component (MNC), degree, edge percolated component (EPC), and centralities such as bottleneck, eccentricity, closeness, and radiality, which can be used to calculate the gene score of PPI network and rank the top 50 genes. According to the gene score, the top ranked genes can be considered as the hub genes. The intersection of these 50 genes from the 7 algorithms revealed the 4 hub genes: fibronectin 1 (FN1), mesothelin (MSLN), plasminogen activator, urokinase (PLAU), and versican (VCAN) (Figure 5(c)).

### 3.6. Survival Analysis

To determine the relationship between hub gene and prognosis, we conducted survival analysis using “survival” of R with clinical information from TCGA database. The optimal cutoff of each gene was determined using the surv_cutpoint function of the survminer package in R. The hub genes were allotted into high and low expression groups based on their respective optimal cutoff values: VCAN (5416), PLAU (1808), MSLN (429), and FN1 (31190). High expression of VCAN (*p* = 0.002), PLAU (*p* < 0.001), MSLN (*p* < 0.001), and FN1 (*p* = 0.004) in PC was related to poor prognosis (Figures 6(a)–6(d)).

## 4. Discussion

Population aging is becoming a major concern, and the rise in incidence of PC [14] has increased the burden on our economy. More emphasis has been laid on improving our understanding of PC pathogenesis and the quest for new treatment alternatives. RNA sequencing technology has been implemented to find DEGs between tumor and normal tissues. In spite of the large number of studies performed till now, there is inconsistency and substantial variation among results due to multiple factors.

The article "Identification of Candidate Therapeutic Target Genes and Profiling of Tumor-Infiltrating Immune Cells in Pancreatic Cancer via Integrated Transcriptomic Analysis" was retracted in 2023. Reasons: suspected computer-generated content; unreliable results or conclusions; concerns about the data; concerns about the results or conclusions.

In our study, we used the RRA method to minimize errors and biases among the 3 datasets. Finally, 350 upregulated and 243 downregulated robust genes were selected. Many of these genes have been reported to be oncogenic, such as gamma-aminobutyric acid type A receptor pi subunit (GABRP) [15], sulfatase 1 (SULF1) [16], and trefoil factor 1 (TFF1) [17]. Interestingly, some of these genes have also been documented as antioncogenes, such as aquaporin 8 (AQP8) [18], glycine N-methyltransferase (GNMT) [19], and zinc transporter ZIP5 (SLC39A5) [20]. In addition, other genes, including follistatin-like 1 (Fstl1), thymosin b10 (TMSB10), and G protein-coupled receptor (GPR87), were obtained. The function of these genes is still unclear, and further research is needed.

Prior studies have shown that TAMs promote tumor occurrence and proliferation and induce immunosuppression [21]. However, the mechanism is still unclear, warranting further research. As antigen-presenting cells, dendritic cells can activate T cells and exert antitumor effects. Dendritic cells exert a vital function in the initial stages of tumor immunity activation [22]. DC maturation is necessary to provide costimulatory signals to T cells, but while resting DCs occur within tumors, it is often insufficient to induce potent immunity, particularly in light of suppressive mechanisms within tumors [23]. Also, Bindea et al. [24], Quail and Joyce [7], and Fridman et al. [25] reported that tumor microenvironment is closely related to the tumorigenesis and tumor progression, as well as resistance to immunotherapy. Based on the cancer-immune cycle theory, antigen-presenting cells capture and process antigens released by cancer cells, and T cell activation exerts an important function in the antitumor process. We may infer that a change in the tumor microenvironment could be related to tumor pathogenesis and immune escape for PC, but this requires further research for substantiation.

To further clarify the functional role of these robust DEGs, we conducted enrichment analyses. GO annotation showed that these DEGs were closely associated with the ECM. Indeed, as we all know, abnormal ECM attachment is an important step in tumorigenesis. The ECM also exerts a vital function in regulating tissue development and homeostasis, and its dysregulation promotes tumor progression [26].

The result of KEGG revealed that abnormal amino acid metabolism and signaling pathways are involved in the pathogenesis of PC. Altogether, these results provide new insights for further studies.

The article "Identification of Candidate Therapeutic Target Genes and Profiling of Tumor-Infiltrating Immune Cells in Pancreatic Cancer via Integrated Transcriptomic Analysis" was retracted in 2023. Reasons: suspected computer-generated content; unreliable results or conclusions; concerns about the data; concerns about the results or conclusions.

In the present study, we also created a PPI network using the STRING database. One key module was identified using the MCODE plugin. Finally, 4 hub genes, including FN1, MSLN, PLAU, and VCAN, were screened, and survival analysis based on hub gene expression was performed with clinical information from TCGA database.

FN1, which can promote the production of stromal components [27], is also involved in cell proliferation and migration [28, 29]. Fibronectin 1 (FN1) has been suggested to be associated with the occurrence of various tumors [30–32]. PC is characterized by abundant tumor stroma fibrosis. However, the exact role of FN1 in the pathogenesis of PC remains blurred. Previously, Han et al. found statistically significant improved survival rates in gastric cancer patients with low FN1 expression [33]. This study result is similar to our findings. We found that FN1 expression in PC tumor tissues was higher, compared with nontumor tissues, and high FN1 expression correlated with a worse prognosis (*p* = 0.004). In addition, higher macrophage infiltration was found in PC tumor tissue compared to normal tissue. The underlying reason may be that the shedding of TAM produces extracellular vesicles (FN1 is one of the main components), reducing pancreatic tumor cell sensitivity to chemotherapy drugs through the ERK pathway [34]. In addition, studies have found that FN1 protein can promote the proliferation of PC cells [35]. High FN1 expression has also been correlated to larger tumor diameter, worse TNM stage, or even more advanced AJCC stage [27].

MSLN was first discovered on the surface of mesothelial cells in 1992 [36]. In subsequent studies, it was found that MSLN may be involved in cell adhesion and differentiation, to name a few [37]. In addition, high MSLN RNA expression correlated with poor prognosis in patients with solid tumors, such as breast cancers [38], ovarian cancers [39], and cholangiocarcinoma [40]. These reports are consistent with our findings. In our study, high mesothelin levels were expressed in PC tissues and high MSLN expression was associated with a poor prognosis. MSLN is overexpressed in some solid tumors and underexpressed in normal tissues, which makes MSLN a potential therapeutic target gene. Excitingly, multicentric clinical trials have already proposed the hypothesis that MSLN could be an important target for immunotherapy [41–43].

Herein, we also found significantly higher PLAU expression levels in PC tissues, which correlated with poor prognosis. PLAU gene can promote the digestion of ECM components. It has been suggested that protein digestion can promote pancreatic ductal metaplasia, one of the causes of PC [44]. PLAU protein can also promote tumor occurrence, tumor cell proliferation, and invasiveness [45]. In addition, inhibiting PLAU expression can inhibit tumorigenesis and reduce resistance to gemcitabine [46].

The article "Identification of Candidate Therapeutic Target Genes and Profiling of Tumor-Infiltrating Immune Cells in Pancreatic Cancer via Integrated Transcriptomic Analysis" was retracted in 2023. Reasons: suspected computer-generated content; unreliable results or conclusions; concerns about the data; concerns about the results or conclusions.

The VCAN protein, as an important ECM component, is closely related to cell adhesion and angiogenesis [47, 48]. Studies have documented the role of VCAN in promoting tumorigenesis, tumor cell proliferation, and distant metastasis [49]. High expression levels of VCAN have also been reported in ovarian, liver, and colon cancer [50–52]. However, to the best of our knowledge, no attempt has been made to explore the role of VCAN in PC. Our study found higher expression levels of VCAN in PC tissues than in normal tissues, which also correlated with a poor prognosis. It has been reported in the literature that VCAN promotes proliferation and invasion by activating the EGFR and NF-*κ*B pathways [53]; however, its role in PC needs more in-depth analysis.

Our study faces some limitations. Further in vivo and in vitro experiments are needed to confirm the significance of the 4 hub genes in PC.

## 5. Conclusions

The integrated transcriptomic analysis was used to provide new insights into PC pathogenesis. We used the RRA method to merge multiple datasets and used the CIBERSORT algorithm to estimate immune cells' infiltration. Enrichment analysis showed that the DEGs were associated with the occurrence and prognosis of PC. Four hub genes, including FN1, MSLN, PLAU, and VCAN, may be considered as novel biomarkers of PC.

## Figures and Tables

**Figure 1:** Study workflow for identification of hub genes and pathways in pancreatic cancer.

**Figure 2:** Heat map of DEGs in pancreatic cancer and normal tissue samples. (a) Heat map of GSE101448, (b) heat map of GSE15471, (c) heat map of GSE62452, and (d) heat map of 20 upregulated and downregulated robust DEGs. The value represented log_2_ fold change (FC), and the positivity or negativity of the values represented up- or downregulation of genes, which were represented by red or green. Red represents a higher expression level, while green represents a lower expression level. DEGs: differentially expressed genes.

**Figure 3:** Enrichment analysis of robust DEGs. (a–d) GO enrichment analyses. (e–h) KEGG pathway enrichment analysis of robust DEGs. DEGs: differentially expressed genes.

**Figure 4:** Immune cell infiltration profiling in pancreatic cancer and normal tissue samples. (a) Bar plot. (b) Heat map. (c) Violin plot.

**Figure 5:** PPI network of DEGs and selection of hub genes from 7 algorithms including MNC, degree, EPC, bottleneck, eccentricity, closeness, and betweenness. (a) PPI network. (b) The key module. (c) Hub genes were selected by the intersection of the top 50 genes. DEGs: differentially expressed genes. PPI: protein-protein interaction.

The article "Identification of Candidate Therapeutic Target Genes and Profiling of Tumor-Infiltrating Immune Cells in Pancreatic Cancer via Integrated Transcriptomic Analysis" was retracted in 2023. Reasons: suspected computer-generated content; unreliable results or conclusions; concerns about the data; concerns about the results or conclusions.

**Figure 6:** Survival analysis. High expression of (a) VCAN, (b) PLAU, (c) MSLN, and (d) FN1 in pancreatic cancer correlated with poor prognosis.

## Data Availability

The datasets supporting the conclusion of this article are included within the article.

## Abbreviations

PC: Pancreatic cancer
DEGs: Differentially expressed genes
RRA: Robust rank aggregation
PPI: Protein-protein interaction
TAM: Tumor-associated macrophages
ECM: Extracellular matrix
FN1: Fibronectin 1
MSLN: Mesothelin
PLAU: Plasminogen activator, urokinase
VCAN: Versican.

## Supplementary Materials

Supplementary 1 Supplementary Table S1: the 564 robust DEGs.

Supplementary 2 Supplementary Table S2: GO enrichment analysis of the 564 robust DEGs.

Supplementary 3 Supplementary Table S3: KEGG enrichment analysis of the 564 robust DEGs.
